RETRACTED

# The Copper Radioisotopes: A Systematic Review with Special Interest to ^**64**^Cu

**DOI:** 10.1155/2014/786463

**Published:** 2014-05-07

**Authors:** Artor Niccoli Asabella, Giuseppe Lucio Cascini, Corinna Altini, Domenico Paparella, Antonio Notaristefano, Giuseppe Rubini

**Affiliations:** ^1^Nuclear Medicine, University of Bari Aldo Moro, Piazza G. Cesare 11, 70124 Bari, Italy; ^2^Nuclear Medicine, University of Catanzaro Magna Graecia, Viale Europa, Localitá Germaneto, 88100 Catanzaro, Italy

## Abstract

Copper (Cu) is an important trace element in humans; it plays a role as a cofactor for numerous enzymes and other proteins crucial for respiration, iron transport, metabolism, cell growth, and hemostasis. Natural copper comprises two stable isotopes, ^63^Cu and ^65^Cu, and 5 principal radioisotopes for molecular imaging applications (^60^Cu, ^61^Cu, ^62^Cu, and ^64^Cu) and in vivo targeted radiation therapy (^64^Cu and ^67^Cu). The two potential ways to produce Cu radioisotopes concern the use of the cyclotron or the reactor. A noncopper target is used to produce noncarrier-added Cu thanks to a chemical separation from the target material using ion exchange chromatography achieving a high amount of radioactivity with the lowest possible amount of nonradioactive isotopes. In recent years, Cu isotopes have been linked to antibodies, proteins, peptides, and nanoparticles for preclinical and clinical research; pathological conditions that influence Cu metabolism such as Menkes syndrome, Wilson disease, inflammation, tumor growth, metastasis, angiogenesis, and drug resistance have been studied. We aim to discuss all Cu radioisotopes application focusing on ^64^Cu and in particular its form ^64^CuCl_2_ that seems to be the most promising for its half-life, radiation emissions, and stability with chelators, allowing several applications in oncological and nononcological fields.

## 1. Introduction

Copper (Cu) is a transition metal with atomic number 29, known since ancient times. It is an important trace element for most organisms in all kingdoms. In humans, copper plays a role as a cofactor for numerous enzymes, such as Cu/Zn-superoxide dismutase, cytochrome c oxidase, tyrosinase, ceruloplasmin, and other proteins, crucial for respiration, iron transport and metabolism, cell growth, and hemostasis [1, 2].

In the last decades, the scientific knowledge and the technological development permitted to overcome the limit of the morphological imaging and to move in the way of biometabolic imaging. This new approach creates further opportunities for clinical research, diseases diagnosis, and treatment. It allows physicians to generate high-resolution images of the human body noninvasively, diagnose illness, and choose treatment regimens based upon them [3].

RETRACTED

New radioisotopes in Nuclear Medicine can be used in their simple form or bound with carrier molecules for the production of complex radiopharmaceutical, creating new opportunities for different metabolic imaging of several organs and systems.

For widespread use in medicine of any radioisotope, two factors are essential: availability of the isotope and a stable and effective mode of binding with an appropriate chemical carrier [4].

Selection of the proper radionuclide in radiopharmaceutical design is critical and depends upon several factors. The half-life of the radionuclide should allow sufficient uptake and distribution to yield considerable contrast and quality images. The energies of the radionuclide emission should be appropriate for proper detection by the equipment, while cost and availability are also important considerations [3].

With the progress in medical sciences, copper has gained a lot of attention.

Natural copper comprises two stable isotopes, ^63^Cu (69.17%) and ^65^Cu (30.83%), and 27 known radioisotopes, five of them are particularly interesting for molecular imaging applications (^60^Cu, ^61^Cu, ^62^Cu, and ^64^Cu), and in vivo targeted radiation therapy (^64^Cu and ^67^Cu) [4].

Copper radionuclides offer a varying range of half-lives and decay modes [3].

## 2. Production of Cu Radioisotopes

One of the major challenges is the production of radionuclides with high specific activity, that is, a high amount of radioactivity with the lowest possible amount of nonradioactive isotopes.

Preparing high specific activity Cu radionuclides is an even bigger challenge, since Cu is ubiquitous in the environment. For all of the Cu isotopes, a noncopper target is used to produce noncarrier-added Cu. In using a target, having a different atomic number, a chemical separation of the copper radionuclide from the target material is possible. In addition, the experimental conditions for preparing the target and separating the copper radionuclides from it must be as metal-free as possible [3].

The following fundamental step is the extraction of each Cu radioisotope from the target, performed using ion exchange chromatography [5].

The two potential ways to produce Cu radioisotopes concern the use of the cyclotron or the reactor. At the state of the art, the cyclotron production is the most studied.

The main characteristics of the Cu radioisotopes of medical interest and their most common ways of production are reported on Table 1.

### 2.1. ^60^Cu

^60^Cu is a *β* ^+^ emitter with decay properties making it possible candidate tracer for positron emission tomography (PET), even it has the disadvantage of *γ* emissions [4]. ^60^Cu is a proton-rich nuclide that decays to its stable Ni isotopes through a combination of positron decay and electron capture processes. It can be produced on a medical cyclotron at relatively low costs using proton or deuteron induced reactions on enriched ^60^Ni targets [5, 6]. Other ways of production have been recently developed (e.g. ^nat^Co + ^3^He, ^nat^Co + a) [7, 8].

RETRACTED

### 2.2. ^61^Cu

^61^Cu isotope can be produced from zinc, nickel, or cobalt targets on a medical cyclotron using proton or deuteron or alpha particles induced reactions. Necessity of highly enriched Ni and Zn targets or high-energy particle beams limited accessibility of ^61^Cu for biomedical use, until more economic production methods from natural Zn or Co will be developed [9, 10]. Half-life longer than that of ^60^Cu and ^62^Cu makes ^61^Cu better choice for prolonged imaging of processes with slower kinetics. This isotope, however, is much less popular in today's biomedical studies than other copper radioisotopes [4, 8, 11–14].

### 2.3. ^62^Cu

^62^Cu has unique properties being almost pure *β* ^+^ emitter (98%) with short half-life of 9.7 min. ^62^Cu is a proton-rich nuclide that decays to its stable Ni isotope through a combination of positron decay and electron capture processes. It can be produced on a medical cyclotron using proton or deuteron induced reactions on enriched ^62^Ni targets. ^62^Cu can also be produced indirectly through its parent ^62^Zn in a ^62^Zn/^62^Cu generator system. This is the preferred option, reducing the levels of radioactivity that need to be manipulated and allowing ^62^Cu to be eluted as required [5].

Current ^62^Zn/^62^Cu generators can start with ^62^Zn activities of 5-6 GBq, 93% of this activity being released as ^62^Cu in the first 3.2 mL of eluate; however relatively short half-life of parent ^62^Zn makes these generators operable for not more than three days.

Currently the proton induced reactions on natural copper is the method of choice for the production of the mother nuclide ^62^Zn. Recently, ^62^Cu production was also investigated via ^nat^Zn + p reactions [15, 16].

This isotope is currently the most intensively studied copper radioisotope besides ^64^Cu [4].

### 2.4. ^64^Cu

^64^Cu is a highly unusual isotope because it decays by three processes, namely, positron, electron capture, and beta decays. This property allows either cyclotron or reactor production, with the latter route resulting in either low specific activity (n,*γ*) or high specific activity (n,p) products [5].

At present, the most common production method for ^64^Cu utilizes the ^64^Ni(p,n)^64^Cu reaction [17, 18].

RETRACTED

The production of noncarrier-added ^64^Cu via the ^64^Ni(p,n)^64^Cu reaction on a biomedical cyclotron was proposed by Szelecsenyi et al. Subsequent studies by McCarthy et al. were performed, and this method is now used to provide ^64^Cu to researchers throughout the United States [17, 19].

The target for producing ^64^Cu is enriched ^64^Ni (99.6%). The ^64^Ni (typically 10–50 mg) is prepared and electroplated onto a gold disk using a procedure modified from Piel et al. [20].

The target is bombarded on the cyclotron. Recently, Obata et al. reported the production of ^64^Cu on a 12 MeV cyclotron, which is more representative of the modern cyclotrons currently in operation [21].

After bombardment, the ^64^Cu is separated from the target nickel in a one-step procedure using an ion exchange column. Typically, 18.5 GBq of ^64^Cu are produced with a 40 mg ^64^Ni target and a bombardment time of 4 h. The specific activity of the ^64^Cu ranges from 47.4 to 474 GBq/*μ*mol (1280 to 12,800 mCi/*μ*mol). The typical yields for ^64^Cu productions are 0.2 mCi/*μ*A·h per mg ^64^Ni. The enriched ^64^Ni can be 85–95% recovered as previously described and reused for future bombardments, which contributes to the cost-efficiency of this method of ^64^Cu production [3].

Another method of  ^64^Cu production is the ^64^Zn(n,p)^64^Cu reaction in a nuclear reactor [22, 23].

Most reactor-produced radionuclides are produced using thermal neutron reactions, or (n,*γ*) reactions, where the thermal neutron is of relatively low energy, and the target material is of the same element as the product radionuclide.

For producing high specific activity ^64^Cu, fast neutrons are used to bombard the target in a (n,p) reaction [22–26].

Unfortunately, one of the byproducts of producing ^64^Cu with a natural Zn target was ^65^Zn (*T* ^1/2^ = 245 d), which limits the practicality of production by this method [27].

Smith et al. separated large amounts of ^64^Cu by product from cyclotron production of ^67^Ga via the ^68^Zn(p,2n)^67^Ga reaction at the National Medical Cyclotron, Sydney, Australia [28]. This method of production has the advantage of being very economical and allows for the production of very large amounts (>111 GBq (>3 Ci)) of reasonably high specific activity material (~31.8 TBq/mmol (~860 Ci/mmol)). The disadvantage is that on-demand production would be problematic, since the major radionuclide produced is long-lived ^67^Ga (*T*_1/2_ = 72 h).

The production of  ^67^Ga, which has identical gamma energies to ^67^Cu, makes activity measurements prior to separation difficult. In addition, isotopes of nickel, cobalt, manganese, and chromium have been observed that while being relatively easy to separate add complexity to the required separation scheme [5].

RETRACTED

Although the proton induced reaction on enriched ^64^Ni plays a key role for practical production, recently the deuteron induced reactions are also intensively studied and seem to be very promising [29].

### 2.5. ^67^Cu

This isotope of copper, owning to interesting decay properties, is potentially useful for radioimmunotherapy, but due to limited availability, researches that actually use this isotope are few, compared to other Cu isotopes [30, 31].

Dynamic growth of radioimmunotherapy can increase demand for this isotope. Medvedev et al. reported an attempt to produce ^67^Cu in a larger scale, which gives perspectives for wider commercial availability of the isotope in the near future [32].

^67^Cu is the longest living copper radioisotope and also one of the most difficult to produce, since it requires fast neutron flux reactor or high-energy proton beams and costly ^68^Zn target [33]. Therapeutic amounts of ^67^Cu can be produced via several reactions on Zn. The production by the reaction ^68^Zn(p,2p)^67^Cu is the largest contributor of ^67^Cu in North America. Providing a reliable supply of ^67^Cu by this method requires dedicated proton beam and chemistry station that are rarely possible at one of these multipurpose facilities [34, 35].

The ^68^Zn(p,2p)^67^Cu reaction requires increasing proton energy, from 20 to 70 MeV, according to Stoll et al. (which includes data from two other studies) [36].

Due to the nature of the spallation process, there will always be a variety of products in the target and enriched targets are seldom used except to determine the reaction cross section. Targets are mainly zinc metal foils which allow for greater heat dissipation and have a higher density than zinc oxide [34, 36].

A small subset of the literature involves the use of a low energy proton beam, 20 MeV, driving a reaction on ^70^Zn(p,a)^67^Cu. The presence of ^67^Ga complicates gamma counting of the sample until after a radiochemical separation. Large amounts of  ^65^Zn are also expected to accumulate in any recycled target due to its 244-day half-life. A demonstration with a larger target mass will determine if this method of production is comparable to other techniques. In contrast to other production methods, the ^70^Zn(p,a)^67^Cu reaction does not coproduce large amounts of other radioisotopes due to the low energy protons used [34, 37].

The production of ^67^Cu in a nuclear reactor by the reaction ^67^Zn(n,p)^67^Cu has been pursued in part due to its simplicity. One only needs to place a suitably contained zinc target in a commercial or research reactor to produce a usable amount of ^67^Cu. However, access to reactors, waste concerns, and undesirable side reactions complicate the use of this reaction for extended productions and medical applications. In the literature the production of ^67^Cu by the reaction ^68^Zn(*γ*,p)^67^Cu is also reported. Linear accelerators producing 30–60 MeV electrons were focused on a convertor plate, usually tungsten or tantalum, which produces photons with a similar energy range [34].

RETRACTED

However, the best yield for the (*γ*,p) reaction on an enriched target only used a few milligrams of zinc; a demonstration with a larger target is required to produce a more accurate yield and validate this method [34].

## 3. Clinical Application

Nuclear medicine imaging provides information about function and structure, using safe, not invasive, and cost-effective techniques for diagnosis and therapy [38].

This discipline is of great importance to medical specialties such as cardiology, neurology, oncology, orthopedics, endocrinology, hematology, nephrology, and pulmonology [38–43].

Copper radioisotopes can have a “conventional role” as radioactive markers that can be added to carrier molecules, conferring all the biological targeting specificity that is needed; furthermore, they can be used as “real tracers,” when directed at the in vivo study of the Cu metabolism itself.

As molecular imaging continues to advance, PET and single photon emission computed tomography (SPECT) techniques are nowadays an integral part of the molecular imaging toolbox; among all the available molecular imaging strategies, PET and SPECT allow targeting of extracellular, cell surface, intracellular proteins, and nucleic acids.

Availability of Cu isotopes for preclinical and clinical research has greatly improved in recent years, also because many potential chelators were developed during over past 20–30 years [4, 44, 45].

The well-established coordination chemistry of Cu allows for its reaction with a wide variety of chelator systems that can potentially be linked to antibodies, proteins, peptides, and other biologically relevant small molecules [3].

Cu metabolism varies from individual to individual. Physiological and pathological conditions that influence Cu metabolism include inherited copper metabolic defects, such as Menkes syndrome and Wilson disease, and acquired copper metabolism disorder or imbalance caused by pregnancy, inflammation, and tumor growth, metastasis, angiogenesis, and drug resistance [46–48].

All Cu radioisotopes are currently investigated for clinical applications but at the state-of- art ^64^Cu, and, in particular, its form ^64^CuCl_2_ seems to be the most promising for its half-life, radiation emissions, and stability with chelators.

RETRACTED

### 3.1. The Role of Cu in Oncology

In the last years, many preclinical studies have demonstrated an effect of Cu on cancer development. In fact, in comparison with normal human subjects, significantly higher copper levels have been measured in serum and tumor cells of patients with cancer including prostate, breast, and brain cancer [49].

^64^CuCl_2_ is the most widely isotope studied, for its potential role in PET imaging and therapy; it has been bound to several carrier that can be applied to monitor copper metabolism status and guide personalized copper chelator treatment in cancer patients [50].

#### 3.1.1. Cu-Labeled Antibodies and Peptides for Tumor Targeting

Monoclonal antibodies (mAbs) are a vast group of biotechnologically produced proteins, with constantly rising number of applications in immunotherapy, targeted drug delivery, and in vivo/in vitro diagnostics. ^64^Cu-labeled antibodies for PET imaging are trastuzumab (breast cancers expressing human epidermal growth factor receptor 2 or HER2), cetuximab (targeting EGFR-epidermal growth-factor receptor expressing tumors), TRC105-Fab (targeting CD105), and etaracizumab (antibody against human *α*_*v*_ *β*_3_ integrin) [4].

Radiolabeling of trastuzumab as well as related fragments and antibodies have been investigated for both diagnostic and radiotherapeutic applications [51].

EGFR expression is increased in many human tumors such as breast cancer, squamous-cell carcinoma of the head and neck, and prostate cancer. At present mAbs, which block the binding of EGF to the extracellular ligand-binding domain of the receptor, have shown promise from a therapeutic standpoint. Cetuximab (C225; Erbitux, Bristol-Myers Squibb, New York, NY) was the first mAb targeted against the EGFR approved by the U.S. Food and Drug Administration (FDA) for the treatment of patients with EGFR-expressing, metastatic colorectal carcinoma [52].

The growth and metastasis of most solid tumors depend on angiogenesis, without which they cannot grow beyond a few millimeters in size. The most widely studied angiogenesis-related targets include CD105 (i.e., endoglin), integrin *α*_*v*_ *β*_3_, and vascular endothelial growth factor receptors (VEGFRs) [53].

CD105 immunohistochemistry is now the accepted standard approach for identifying actively proliferating tumor vessels; it has several advantages over the other targets, including high levels of expression in a wide variety of solid malignancies, independence from its expression on neoplastic cells, lack of tumor histotype specificity, and immediate accessibility of malignant lesions through the bloodstream. With high affinity/specificity for CD105, radiolabeled TRC105-Fab demonstrated its potential in several preclinical tumor models to serve as a promising diagnostic agent for PET imaging. [54].

RETRACTED

#### 3.1.2. Cu Labeled Peptides for Tumor Angiogenesis

^64^Cu labeled peptides for targeted cancer therapy/imaging are one of the largest groups of copper radiopharmaceuticals currently researched. They are built of a targeting peptide such as bombesin or octreotide analogue, a linker, and a bifunctional chelator (BFC), commonly tetraazamacrocycle derivate, like TETA or DOTA. The peptide binds to a specific receptor expressed by cancer cells, while copper isotope-BFC moiety allows localization of the tumor by positron emission detection. Attractiveness of peptides for targeted radiotherapy, in comparison to monoclonal antibodies, comes from their good tissue distribution, fast clearance, low immunogenicity, and inexpensive, automated production [4].

It was also observed that copper salts were the simplest angiogenic component of the tumor extract, acting through a stimulation of the migration of the endothelial cells [49].

Alpha *v* beta 3 (*α*_*v*_ *β*_3_) is one of the most widely studied integrins, since it is upregulated in endothelial cells involved in active angiogenesis but not in quiescent endothelial cells, making it an ideal biomarker for angiogenesis and tumor imaging. Tumors where *α*_*v*_ *β*_3_ is found to be highly expressed include glioblastomas, breast and prostate tumors, malignant melanomas, and ovarian carcinomas. The *α*_*v*_ *β*_3_ integrin binds to extracellular proteins through a specific binding pocket that recognizes the three-amimo-acid sequence, arginine-glycine-aspartic acid (Arg-Gly-Asp or RGD).

Sprague et al. conjugated c (RGDyK) to a different chelator, CB-TE2A, and found that the corresponding ^64^Cu complex was taken up specifically by osteoclasts, which are upregulated in osteolytic lesions and bone metastases. These investigations open the possibility of other applications for imaging *α*_*v*_ *β*_3_ in diseases, such as osteoarthritis or osteoporosis, as well as imaging osteolytic bone metastases [52, 54].

Hao et al. found ^61^Cu-1,4,7,10-tetraazacyclododecane-1,4,7,10-tetraacetic acid (DOTA)-human serum albumin to be good blood pool imaging agent and suggested its application in antiangiogenic therapy monitoring [55].

^67^Cu is one of the best-suited isotopes for radioimmunotherapy, because its half-life is long enough to allow good biodistribution within tumor (similar to biological half-life of many mAbs), relatively low gamma radiation abundance (lower whole body dose for patient and safer for medical personnel), higher tumor uptake (compared to iodine-131), and simple radiolabeling procedure. Examples of ^67^Cu labelled mAbs are chCE7, an anti-L1-cell adhesion molecule antibody for neuroblastoma, ovarian, and some renal carcinoma therapy, Lym-1 for non-Hodgkin's lymphoma, C595 an anti-MUC1 mucin antibody for bladder cancer treatment [4].

RETRACTED

#### 3.1.3. Cu Labeled Somatostatin Analogs for Targeting Neuroendocrine Tumors

Somatostatin is a 14-amino-acid peptide involved in the regulation and release of several hormones.

Somatostatin receptors (SSRs) are present in many different normal organ systems, such as the central nervous system (CNS), the gastrointestinal tract, the exocrine, and endocrine pancreas, breast, and lung, making it a viable disease target [52].

Targeting of SSRs in tumors has been a goal in cancer treatment and diagnosis since the 1980s, labeling octreotide (OC) with 123I, 111In, and ^67^Ga [52].

In the first-in-humans study, Pfeifer et al. found ^64^Cu-DOTATATE PET useful for clinical somatostatin receptor imaging. Compared with ^111^In-DTPA-octreotride SPECT, ^64^Cu-DOTATATE PET provided superior image quality, detected more true-positive lesions, and was associated with a lower radiation burden [56].

#### 3.1.4. Imaging Tumor Hypoxia

It is well established that hypoxia is an important determinant of the overall tumor response to conventional therapy. Hypoxia can result in an increase in tumor aggressiveness, failure of local control, and activation of transcription factors that support cell survival and migration [57].

The ability to locate and quantify the extent of hypoxia within solid tumors by using noninvasive nuclear imaging would facilitate early diagnosis and help clinicians select the most appropriate treatment for each individual patient [52].

Diacetyl-2,3-bis(N^4^-methyl-3-thiosemicarbazone) (ATSM) seems to be an innovative compound for hypoxia imaging which could be labeled with copper positron emitter radioactive isotopes like ^60/61/62/64^Cu. The metabolism and pharmacological pathway of Cu-ATSM complex is the same for all the copper isotopes, and the choice for clinical use between these isotopes is based on physical properties. ^60^Cu-ATSM was clinically studied for monitoring tumor hypoxia in lung and cervical cancer and found to be feasible for prediction of tumor response to therapy [57, 58]. Chao et al. suggested that PET images obtained with ^60^Cu-ATSM can be used for intensity-modulated radiation therapy of head and neck cancer [59].

^61^Cu-2-acetylpyridine thiosemicarbazone (^61^Cu-APTS) complex, for PET imaging of cancer, was proposed by Belicchi-Ferrari et al. Using APTS as a ligand can give additional antiproliferative activity to the compound, which was previously observed by other authors [60].

^62^Cu-pyruvaldehyde-bis(N^4^-methylthiosemicarbazone) (^62^Cu-PTSM) can be used together with ^62^Cu-ATSM to obtain complementary data on tumor hypoxia and blood circulation in a single PET session [4, 61].

^64^Cu presents the best compromise between adapted physical properties (sufficiently long half-life, better intrinsic image resolution with low *β* ^+^ maximal energy) and good production yield (reasonable production costs) [57].

RETRACTED

Similar to ^60/61/62^Cu isotopes, ^64^Cu-ATSM is subject of many ongoing researches as selective tumor hypoxia imaging agent. Phase II clinical trials of  ^64^Cu-ATSM PET/CT are monitoring therapeutic progress in patients with cervical cancer. Similar compound, ^64^Cu-diacetyl-bis(N^4^ ethylthiosemicarbazone) (^64^Cu-ATSE), has wider tissue-oxygenation level specificity than ^64^Cu-ATSM. In various clinical trials, ^64^Cu-ATSM provided images of tumor hypoxia that improved the clinical outcome of patients submitted to external beam radiotherapy [57].

In conclusion, ^64^Cu-ATSM has several advantages over other radiopharmaceuticals used for PET of hypoxia, including a simple and rapid method for radiolabeling, faster clearance from normoxic tissues (allowing a short time between injection and imaging), a simple method for quantification, and very good image quality [57].

#### 3.1.5. Chemotherapy Resistance

The chemotherapeutic agent Cisplatin (DDP) is a highly polar molecule not readily diffusible across lipid membranes. In many cell types, DDP triggers, as the Cu, a rapid degradation of human copper transporter 1 (hCtr1). This DDP action is obtained at much lower concentrations and more rapidly respect to copper. hCtr1 expression decreases with the acquisition of a DDP resistance, so, in accordance with this phenomenon, a reduced Cu intracellular uptake should be observed in presence of a DDP resistance [49].

In particular, ^64^CuCl_2_ can be used to test the drug resistance to therapeutic schemes based on DDP, as in patients affected by breast, ovarian, or colon cancer [49].

#### 3.1.6. Prostate Cancer

In view of the fact that human tumor tissues contain high concentrations of copper, Peng et al. hypothesized that human prostate cancers express high levels of hCtr1 and can be detected by ^64^Cu PET. hCtr1 is a high-affinity copper transporter that mediates cellular uptake of copper in humans and is highly expressed in the liver [62].

The hCtr1 expression level may be related to the aggressiveness or prognosis of the prostate cancer and to the response of prostate cancer to cisplatin chemotherapy because hCtr1 was recently reported to be able to mediate cellular uptake of cisplatin [62].

RETRACTED

On the ^64^Cu PET images, there was less background activity in the urinary bladder region because ^64^CuCl_2_ was cleared mainly by the hepatobiliary pathway, instead of renally as ^18^F-FDG [62].

### 3.2. The Role of Cu in Neurology

It was assumed that Wilson Disease (WD) patient will have increased uptake of copper in brain tissue and pathologic analysis of the brain may show gliosis and neuronal loss in association with increased Cu deposition. Some WD patients have copper accumulation in the brain and show neurological disorder, while others do not [63].

Diagnosis of WD can be challenging as symptoms mimic other diseases and may gradually appear over time. In addition, the presence of many different mutations in Atp7b gene makes it difficult to screen and diagnose WD by genetic testing. ^64^CuCl_2_ PET may change the management of WD patients because it could reflect the symptoms variation of WD and thus affect the treatment strategy. With more detailed information and a SUV cut-off value obtained from further validation of the methodology, ^64^CuCl_2_ PET could serve as a simple, straightforward, and noninvasive method for WD diagnosis [63].

Diagnosis of Alzheimer's disease has been investigated using imaging agent that targets *β* amyloid plaque burden, but new approach highlights altered copper homeostasis. A bis-(thiosemicarbazonato) complex radiolabeled with ^64^Cu can be used for a new and alternative method for the noninvasive diagnosis of Alzheimer's disease using PET. This approach has the potential to offer complementary information to other diagnostic procedures that elucidate plaque burden [64].

Furthermore, studies in Parkinson's patients and cerebral perfusion preclinical studies have been performed in freely moving subjects using ^60/61/62/64^Cu-PTSM and later ^62^Cu-ethylglyoaxal bis(thiosemicarbazone) (^62^Cu-ETS), suggesting their potential application to clinical neurology or neuropsychiatry [65–68].

### 3.3. Other Potential Roles

Studies over the last 20 years investigated the usefulness of Cu radioisotopes complexed with ATSM for the detection of myocardial perfusion. ^62^Cu-ATSM complex is widely researched for PET imaging of myocardial ischaemia; ^64^Cu-ATSM seems to be useful to study myocardial hypoxia [69–72].

Furthermore, 5,13-dioximino-6,9,9,12-tetramethyl-7,11-diazaheptadeca-6,11-diene complex of ^64^Cu synthesized by Packard et al. can be potentially used as myocardial perfusion imaging agent and PECAM-1 antibody conjugated with DOTA and labeled with ^64^Cu was successfully performed to evaluate induced myocardial infarction in mouse model [70].

RETRACTED

Novel approach for therapy of multinodular goitre, using human chorionic gonadotropin (hCG) directly labeled with ionic Cu *β* ^+^ emitters was proposed by Maiti et al. [73]. Initial studies indicate that copper-hCG complex half-life is shorter than that of a hCG-TSH (thyroid stimulating hormone) receptor complex, thus hyperactive thyroid cells can be destroyed before internalization of the receptor occurs. More in vitro and in vivo studies are required to assess usefulness of this purpose [4].

Interesting perspectives for copper imaging with PET could be related to the analysis of inflammatory conditions [49].

Nanoparticles labeled with ^64^Cu were used to detect macrophages in atherosclerotic plaques showing high sensitivity and direct correlation with CD68 expression [74].

Locke et al. showed in mouse model that ^64^Cu labeled peptides targeting the formil peptide receptor on neutrophil in vitro accumulate at sites of inflammation in vivo, suggesting that new radiolabeled peptides may prove to be a useful tool to probe inflammation [75].

## 4. Conclusions

Copper isotopes are gaining a worthy role in the PET radionuclide scenario. Versatility of copper isotopes gives them a strong position in development of new pharmaceuticals. Currently, there are few applications in medicine but numerous ongoing studies will most likely result in novel use in the future.

The longer half-life allows ^64^Cu to be produced at regional or national cyclotron facilities and distributed to local nuclear medicine departments. In addition, ^64^Cu longer half-life is compatible with the time scales required for the ability to create complex radiopharmaceutical, optimal biodistribution of slower clearing agents, such as monoclonal antibodies (mAbs), nanoparticles, and higher molecular weight polypeptides requiring longer imaging times allowing several applications in oncological and nononcological fields.

## Figures and Tables

**Table 1:** Main characteristic of the medically relevant Cu radioisotopes.

Isotope	*T*_1/2_	Decay mode	Energy (keV)	Production			
					Incident beam energy (MeV)	Reaction	Yield at recovery (MBq/*μ*Ah or MBq/mg)
^ 60^Cu	23.7 min	*β* ^+^ (93%)	2940	Cyclotron	11	^60^Ni(p,n)^60^Cu	370
		*γ* (7%)	511/467/826/1332				

^ 61^Cu	3.32 h	*β* ^+^ (60%)	1159	Cyclotron	19	^61^Ni(p,n)^61^Cu	573**
		*γ* (40%)	511/283/589/656				

^ 62^Cu	9.7 min	*β* ^+^ (98%)	2925	Cyclotron	5–14	^62^Ni(p,n)^62^Cu	19800**
		*γ* (2%)	511				

^ 64^Cu	12.7 h	*β* ^+^ (19%)	657	Cyclotron	12	^ 64^Ni(p,n)^64^Cu	243***
		*γ* (43%)	511/1346		19	^ 64^Ni(d,2n)^64^Cu	388***
		*β* ^−^ (38%)	141		ND	^ nat^Zn(p,xn)^64^Cu	67
				Reactor	1.8*	^ 64^Zn(n,p)^64^Cu	14.5****
					ND	^ 63^Cu(n,*γ*)^64^Cu	ND

^ 67^Cu	61.83 h	*β* ^−^ (100%)	390/482/575		ND	^ 68^Zn(p,2p)^67^Cu	ND
		*γ* (52%)	91/93/185	Cyclotron	ND	^ 70^Zn(p,a)^67^Cu	ND
					ND	^ 67^Zn(n,p)^67^Cu	ND
					ND	^ 68^Zn(g,p)^67^Cu	ND

ND: data not available.

RETRACTED

*Approximate minimum neutron energy.

**Predicted yield.

***Maximum of results.

****Mean of results.
